The article "A Comparative Analysis of Machine Learning Algorithms to Predict Alzheimer's Disease" was published in 2021. Journal: J Healthc Eng.

# A Comparative Analysis of Machine Learning Algorithms to Predict Alzheimer's Disease

**DOI:** 10.1155/2021/9917919

**Published:** 2021-07-02

**Authors:** Morshedul Bari Antor, A. H. M. Shafayet Jamil, Maliha Mamtaz, Mohammad Monirujjaman Khan, Sultan Aljahdali, Manjit Kaur, Parminder Singh, Mehedi Masud

**Affiliations:** ^1^Electrical and Computer Engineering Department, North South University, Dhaka 1229, Bangladesh; ^2^Department of Computer Science, College of Computers and Information Technology, Taif University, P O. Box 11099, Taif 21944, Saudi Arabia; ^3^Computer Science Engineering, School of Engineering and Applied Sciences, Bennett University, Greater Noida 201310, India; ^4^School of Computer Science and Engineering, Lovely Professional University, Phagwara, India

## Abstract

Alzheimer's disease has been one of the major concerns recently. Around 45 million people are suffering from this disease. Alzheimer's is a degenerative brain disease with an unspecified cause and pathogenesis which primarily affects older people. The main cause of Alzheimer's disease is Dementia, which progressively damages the brain cells. People lost their thinking ability, reading ability, and many more from this disease. A machine learning system can reduce this problem by predicting the disease. The main aim is to recognize Dementia among various patients. This paper represents the result and analysis regarding detecting Dementia from various machine learning models. The Open Access Series of Imaging Studies (OASIS) dataset has been used for the development of the system. The dataset is small, but it has some significant values. The dataset has been analyzed and applied in several machine learning models. Support vector machine, logistic regression, decision tree, and random forest have been used for prediction. First, the system has been run without fine-tuning and then with fine-tuning. Comparing the results, it is found that the support vector machine provides the best results among the models. It has the best accuracy in detecting Dementia among numerous patients. The system is simple and can easily help people by detecting Dementia among them.

## 1. Introduction

Machine learning (ML) is defined as the study of computer programs that leverage algorithms and statistical models to learn through inference and patterns without being explicitly programmed [1]. ML algorithms learn over experience and improve automatically. It finds techniques, trains models, and uses the learned approach to determine the output automatically [2]. Machine learning systems can also adjust themselves to a changing environment.

A model is a machine learning system that has been trained to identify specific types of patterns using an algorithm in a machine learning system [3]. That means it processes the data and finds out the hidden structures in a dataset [4]. The feature extraction and the known answers of a dataset determine the formula that relies upon the input and output functions and applies it to new data to predict the response [5]. Hence, the model's algorithm uses a collection of data for training and builds a way to predict the output and saves that procedure for future purposes.

The article "A Comparative Analysis of Machine Learning Algorithms to Predict Alzheimer's Disease" was published in 2021. Journal: J Healthc Eng.

A support vector machine (SVM) is a supervised machine learning model that uses classification algorithms for two-group classification problems. Support vector machine is a fast and dependable classification algorithm that performs very well with a limited amount of data to analyze [6]. SVMs are a group of similar supervised learning techniques that are used for classification and regression problems [7].

The logistic regression model is the appropriate regression analysis. Logistic regression is predictive regression analysis [8]. To classify data and to illustrate the relationship between one dependent binary variable and one or more independent nominal, ordinal, interval, or ratio-level variables, logistic regression is used [9].

In a machine learning system, a decision tree algorithm partitions the data into subsets. A decision tree's purpose is to sum up the training data in the smallest tree possible [10]. The decision tree is a supervised classification method that carries out a split test in its internal node and forecasts an example target class in its leaf node [11]. Decision tree algorithms are used to classify the characteristics to be evaluated at any node to specify the “best” splitting [12]. Decision trees are commonly used in classification problems because of their versatility and consistency.

The random forest is a supervised learning algorithm. Random forest is a versatile, easy-to-use machine learning algorithm that provides, most of the time, a fantastic result even without hyperparameter tuning [13]. Its simple design and variety are also some of the most used algorithms [14].

SVM can be applied to nonlinear problems, whereas logistic regression can only work with linear ones. SVM operates outliers better, as it derives maximum margin solution. Decision trees are better at dealing with collinearity than logistic regression. For categorical values, decision trees outperform logistic regression. A random forest is a set of decision trees that are randomly generated, and the expected output is chosen by the forest's majority vote. Decision trees are less reliable and accurate than random forest. SVM solves nonlinear issues using kernel methods, whereas decision trees apply hyperrectangles in input space to solve the problem. For a classification problem, SVM performs better than random forest [15].

The article "A Comparative Analysis of Machine Learning Algorithms to Predict Alzheimer's Disease" was published in 2021. Journal: J Healthc Eng.

Machine learning models are now widely used in medical diagnosis [16–19]. This paper compares different machine learning performances to diagnose Alzheimer's syndrome. Alzheimer's syndrome is an inherited, irreversible brain condition that steadily affects the ability to perform the necessary things, memory, and reasoning skills [20]. A massive proportion of neurons stop working in Alzheimer's disease, losing synaptic connections [21]. Alzheimer's diseases are infrequent in people aged between their 30s and mid-60s [22]. Symptoms can include a shift in sleep habits, depression, anxiety, and difficulties doing basic tasks such as reading or writing and aggressive actions, and poor decision-making also happened in Alzheimer's disease [23]. Alzheimer's disease and initial changes in the brain begin 10–20 years before the onset of symptoms [24]. It progressively leads to memory damage and decreases thinking abilities [25]. The leading cause of this disease is Dementia. A report shows that around 40–50 million people worldwide are suffering from Dementia, and this number will be increased to around 131.5 million by 2050 [26]. Approximately 70% of people who have Dementia are from low-income countries; see Figure 1.

Dementia is the failure of brain function, understanding, recognizing, thinking, and behavioral skills to such a level that an individual faces problems in everyday life and behaviors [28]. Few people with Dementia are unable to deal with their emotions, and their personalities can be changed [29]. From the mildest stage, Dementia varies in severity [30]. It mainly affects older people. No cure is available other than treatment [31].

There is little data available on Alzheimer's patients in Bangladesh. According to the WHO data published in 2017, Alzheimer's or Dementia deaths in Bangladesh reached 9,917 or 1.26% of the total deaths, which was the last data found in this aspect that ranks Bangladesh number 152 globally [32]. In Bangladesh, the awareness about Alzheimer's is now in the primary stage. Therefore, impacted patients and families are regularly experiencing various issues [33]. The fund for researching Alzheimer's is limited. A lower-middle-income country like Bangladesh is not yet prepared for the management of Alzheimer's [34]. Besides that, almost one-fifth of the Bangladeshi adult population is overweight, according to a global study [35], which is the leading risk factor for Alzheimer's. Therefore, there are more chances of occurrences of Alzheimer's [36]. To give a treatment for this disease, physicians tend to test individuals for Alzheimer's disease by obtaining a medical and family history and psychiatric history from the point of view of specialists such as neurologists, neuropsychologists, geriatricians, and geriatric psychiatrists [37].

The article "A Comparative Analysis of Machine Learning Algorithms to Predict Alzheimer's Disease" was published in 2021. Journal: J Healthc Eng.

Studies show that the situation may improve if people can detect Alzheimer's disease early by taking therapy at the initial stage [38]. For this, they have to predict the progress of the disease accurately from mild condition to Dementia. Machine learning technology can help to predict accurately early Alzheimer's disease. There are many machine learning systems, but they give inconsistent and inaccurate predictions. They also have overfitting and underfitting issues. Therefore, a model has been developed by us which can indicate Alzheimer's disease early, using machine learning to support medical technicians. It will verify and show if anyone has Alzheimer's disease or not.

The remainder of the paper is organized as follows: Section 2 discusses methods and methodology, and Section 3 provides the results and analysis. Finally, in Section 4, the conclusion of the presented work is provided.

## 2. Methods and Methodology

In this section, all methods and materials, the dataset feature's description, block diagram, flow diagram, and evaluation matrices of the system are discussed.

### 2.1. Dataset

The main goal of the system is to predict Dementia in different patients based on various attributes. The longitudinal Magnetic Resonance Imaging (MRI) data from OASIS [39] has been used for the development of the system. The OASIS dataset has a dimension of 373 rows x 15 columns, which is relatively small in the field of machine learning.  Table 1 shows eight different attributes: gender (M/F), person's age (age), years of education (EDUC), socioeconomic status (SSE), mini-mental state examination (MMSE), estimated total intracranial volume (eTIV), normalized whole brain volume (nWBV), and Atlas scaling factor (ASF) have been considered for the final outcome. For range values, a standardization method has been applied for scaling the dataset. A standard score is the number of standard deviations by which the value of a raw score is above or below the mean value of what is being observed or measured. The formula is as follows: *z* = (*x* − *μ*)/*σ*. Here, *µ* is the mean, and *σ* is the standard deviation.

Table 2 shows the eight features of the dataset which have been considered for the proposed model to predict Alzheimer's disease and the description of the features. Most of the features are numerical. Group, hand, and M/F are categorical. All of these terms describe the patient's condition and aid in determining the stage of Dementia using the ML system.

The article "A Comparative Analysis of Machine Learning Algorithms to Predict Alzheimer's Disease" was published in 2021. Journal: J Healthc Eng.

### 2.2. Block Diagram

Figure 2 shows the block diagram of the machine learning system. The OASIS dataset has been used in the system, which contains all the attributes and values. First, the dataset has been analyzed by us for any categorical values, and there are several categorical values present in the dataset. Among them, gender and group attribute columns are converted into numeric values 0 and 1. The correlation between attributes has been checked by us using the “correlation matrix” function based on group attributes and plotted to understand them better. Gender, SES, and ASF showed a closer correlation with the group attribute. After that, the dataset is checked for any null or missing values. SES and MMSE columns have 19 and 2 missing values, respectively. As mentioned earlier, the SES feature has a close correlation with the target attribute. For that reason, the missing values of those rows were not deleted. Instead, the median value is used to fill in those missing values for both features.

Next, the features have been assigned to make the prediction, and the target value has been set so that the model can predict. Then, the dataset was split for training-validation and testing. Random sampling has been used for the split, but this creates an imbalance between training and testing split. So, stratified sampling has been applied with a training-validation size of 80% and a testing size of 20%. After that, standardization has been applied to do the scaling of the features. Furthermore, some histograms and scatterplot visualization have been done on the training split to understand the scenario better. Then the training of this system began. All of the models have been implemented using the scikit-learn library.

### 2.3. Flowchart Diagram

#### 2.3.1. SVM Flowchart

Figure 3 shows the flow diagram of the whole SVM model. First, the support vector machine has been implemented without any fine-tuning. Without fine-tuning, SVM takes regularization parameter *C* as 1, and, for the kernel, it uses the radial basis function (RBF). After that, the grid search has been applied to fine-tune the model. Then, different regularization parameters have been taken for the parameter combinations, such as values *C*, gamma values, and four types of kernels: the RBF, linear, poly, and sigmoid kernel. Also, 5-fold cross-validation has been applied to evaluate all possible combinations. Then, the model was trained again, and there was a significant improvement. The confusion matrix has been calculated based on this version.

#### 2.3.2. Logistic Regression Flowchart

Figure 4 shows the flow diagram of the whole logistic regression model. The same approach has been applied with the logistic regression model, just like the SVM. It determines the independent and dependent variables. It uses the sigmoid function for predicting probabilities and making decision boundaries. The only difference is that the l2 penalty and different regularization parameter values *C* have been used for the fine-tuning.

The article "A Comparative Analysis of Machine Learning Algorithms to Predict Alzheimer's Disease" was published in 2021. Journal: J Healthc Eng.

#### 2.3.3. Decision Tree Flowchart

Figure 5 shows the flow diagram of the whole decision tree model. In the decision tree model, the same approach is followed. The model has been trained without fine-tuning and then used the grid search to find the best parameter values to fine-tune the model. Here, the Gini criterion has been considered a fixed value to evaluate the tree's quality and choose a range of 1 to 10 to evaluate the depth of the tree. It decides every node and goes more in depth. After analyzing all the nodes' choices, it predicts the results for the best solution.

#### 2.3.4. Random Forest Flowchart

Figure 6 shows the flow diagram of the whole random forest model. It is a collection of some decision trees. The process is the same as the decision tree. It preprocesses the data and selects some random samples from the dataset for training. For every selected sample, it forms a decision tree. First, the random forest model has been trained without fine-tuning. Then, just like the SVM, grid search has been used with 5-fold cross-validation and different parameter combinations such as the number of trees in the random forest (n_estimators), what function to use for the number of features to consider at every split, levels in the tree, and method of selecting samples for training each tree. To measure the quality of the tree, the Gini criterion has been used. The entropy criterion has also been tried in the model, but Gini criterion provides better accuracy.

### 2.4. Evaluation Matrices

Figure 7 shows the diagram of the confusion matrix. The confusion matrix is a performance evaluator for the classification models of machine learning. To evaluate the performance of all the developed models, the confusion matrix has been used. The confusion matrix represents how many times our models predict correctly and how many times they predict incorrectly. It categorized the correctly predicted values as true positives and true negatives and also categorized the wrongly predicted values as false positives and false negatives. After organizing all the predicted values in the matrix, the model's performance has been measured through accuracy, precision-recall trade-off, and AUC.

## 3. Results and Analysis

The models' functions, model predictions, analysis, and final results are discussed in this section.

The article "A Comparative Analysis of Machine Learning Algorithms to Predict Alzheimer's Disease" was published in 2021. Journal: J Healthc Eng.

### 3.1. Data Visualization

#### 3.1.1. Histogram

Figure 8 shows the histogram of the training and validation set. Histogram portrays the ratios of the dataset. From the M/F plot, it has been observed that the male-female ratio in the dataset is 60% to 40%. All patients' age in the dataset is 60+ years. The majority of SES is 2, and MMSE is 30. Most of the patients' education years are 12.5. Also, the eTIV, nWBV, and ASF are relatively high.

#### 3.1.2. Correlation Matrix

Figure 9 shows the correlation matrix of the features in the dataset. The correlation matrix indicates how features are interrelated with each other. The group is the main target feature for detecting Dementia. If the value of the group is greater than 0.5, the patients have Dementia. From the correlation matrix, it has been observed that the higher the value of ASF and SES, the more the chances of getting Dementia. It is also observed that males have more chance of getting Dementia than females.

### 3.2. Model

#### 3.2.1. SVM Model

Figure 10 shows the SVM model's prediction before fine-tuning. The predicted result is shown in the confusion matrix, and the model's calculated performance has also been demonstrated. The number of correct predictions is 56, and the number of wrong predictions is 19. It has 85% training accuracy and 74% testing accuracy. It also possesses 59% test recall and 74% test AUC.

#### 3.2.2. SVM Model after Fine-Tuning

Figure 11 shows the SVM model's prediction after fine-tuning. After fine-tuning, the obtained result has improved quite significantly. The SVM model gives 69 correct predictions and only 6 wrong predictions with 92% accuracy. For classification problems, SVM always provides the best accuracy among other models. It gives the best true negative results in the system. It also possesses 91% of both test recall and test AUC. No overfitting or underfitting issues have been observed from the model.

#### 3.2.3. Logistic Regression Model

Figure 12 shows the logistic regression model's prediction before fine-tuning. The confusion matrix shows the actual predicted values using this model. The model gives 56 correct predictions and 19 wrong predictions with 74.7% accuracy. It has given the same accuracy as before fine-tuning by the SVM model. It also holds 70% test recall and 74% test AUC.

#### 3.2.4. Logistic Regression Model after Fine-Tuning

Figure 13 shows the logistic regression model's prediction after fine-tuning. After fine-tuning, the logistic regression model remained the same. The model's results have not changed. It gives the same correct and wrong predictions as before with 74.7% accuracy. No overfitting issue has been detected in the model.

The article "A Comparative Analysis of Machine Learning Algorithms to Predict Alzheimer's Disease" was published in 2021. Journal: J Healthc Eng.

#### 3.2.5. Decision Tree Model

Figure 14 shows the decision tree model's prediction before fine-tuning. The decision tree model gives 56 correct predictions and 19 wrong predictions, the same as the logistic regression model. It offers 100% training accuracy and 72% testing accuracy. It also provides 67% test recall and 71% test AUC.

#### 3.2.6. Decision Tree Model after Fine-Tuning

Figure 15 shows the decision tree model's prediction after fine-tuning. After fine-tuning, the decision tree model has improved quite a lot. It gives 60 correct predictions and 15 wrong predictions with 80% accuracy. It also gives the best true positive results in the system. The least overfitting issue has been experienced in the model.

#### 3.2.7. Random Forest Model

Figure 16 shows the random forest model's prediction before fine-tuning. The random forest model gives 61 correct predictions and 14 wrong predictions. It offers 100% accuracy in training and 81% accuracy in test validation. It also gives 70% recall and 81% AUC on validation.

#### 3.2.8. Random Forest Model after Fine-Tuning

Figure 17 shows the random forest model's prediction after fine-tuning. After fine-tuning, the accuracy of the random forest model decreases. It gives 60 correct predictions and 15 wrong predictions with 80% accuracy. Actually, it has quite similar result to the previous one. Too many overfitting issues have been found in the model.

### 3.3. Model Comparison

#### 3.3.1. ROC and AUC

Figure 18 shows the plotting of receiver operating characteristic (ROC) and comparison of AUC. Since this is a classification problem, the evaluation metrics used in this system were as follows: accuracy, recall, area under the curve (AUC), and confusion matrix. After compiling the results from all the models, it is evident that support vector machine (SVM), more specifically support vector classifier, gave the best overall result in all metrics. However, the decision tree classifier gave the best true positive result. For fine-tuning, grid search has been used in the models. So, the results obtained are the best possible result for the particular dataset. Some overfitting has been noticed in decision tree and random forest models.

#### 3.3.2. Comparison Table

Table 3 shows the comparison table of the models. The table clearly indicates that SVM is the best model among the other models in the system. It has better accuracy, recall, area under the curve, and *F*1 score.

## 4. Conclusion

The main aim of the system is to predict Alzheimer's disease. For predicting Alzheimer's disease or Dementia in adult patients, the “MRI and Alzheimer's” dataset has been used, which has been provided by the Open Access Series of Imaging Studies (OASIS) project. The dataset has been visualized and filled in the missing values. Data has been preprocessed by removing some unnecessary features. The values were standardized to make sure that they easily fit in the ML models. Then the dataset has been used to train SVM, logistic regression, decision tree, and random forest models. For evaluation metrics, accuracy, recall, AUC, and confusion matrix have been used. To improve the system result, the grid search method has been used to fine-tune all developed models. For this particular dataset, the system got the best result using SVM. A more complex model like the random forest classifier suffered from an overfitting issue. For deployment, the SVM model has been used for the best results among all the models. In the future, the system models could be improved by using a larger dataset and more ML models such as AdaBoost, KNN, Majority Voting, and Bagging. This will increase reliability and enhance the performance of the system. The ML system can help the general public get an idea about the possibility of Dementia in adult patients by simply inputting MRI data. Hopefully, it will help patients to get early treatment for Dementia and improve their life.

The article "A Comparative Analysis of Machine Learning Algorithms to Predict Alzheimer's Disease" was published in 2021. Journal: J Healthc Eng.

## Figures and Tables

**Figure 1:** Number of people with Dementia in millions [27].

**Figure 2:** Block diagram.

**Figure 3:** Flowchart of SVM.

**Figure 4:** Flowchart of logistic regression.

**Figure 5:** Flowchart of decision tree.

**Figure 6:** Flowchart of random forest.

**Figure 7:** Diagram of confusion matrix.

**Figure 8:** Histogram of training and validation set.

**Figure 9:** Correlation matrix.

**Figure 10:** SVM model.

**Figure 11:** SVM model after fine-tuning.

**Figure 12:** Logistic regression model.

**Figure 13:** Logistic regression model after fine-tuning.

**Figure 14:** Decision tree model.

**Figure 15:** Decision tree model after fine-tuning.

**Figure 16:** Random forest model.

**Figure 17:** Random forest model after fine-tuning.

**Figure 18:** Plotting of ROC and comparison of AUC.

**Table 1:** OASIS dataset of proposed machine learning system.

Subject ID	MRI ID	Group	Visit	MR delay	M/F	Hand	Age	EDUC	SES	MMSE	CDR	eTIV	nWBV	ASF
OSA2_0001	OSA2_0001_MR1	Nondemented	1	0	M	R	87	14	2.0	27.0	0.0	1987	0.696	0.883
OSA2_0001	OSA2_0001_MR2	Nondemented	2	457	M	R	88	14	2.0	30.0	0.0	2004	0.681	0.876
OSA2_0002	OSA2_0001_MR1	Demented	1	0	M	R	75	12	NaN	23.0	0.5	1678	0.736	1.046
OSA2_0002	OSA2_0001_MR2	Demented	2	560	M	R	76	12	NaN	28.0	0.5	1738	0.713	1.010
OSA2_0002	OSA2_0001_MR	Demented	3	1895	M	R	80	12	NaN	22.0	0.5	1698	0.701	1.034

The article "A Comparative Analysis of Machine Learning Algorithms to Predict Alzheimer's Disease" was published in 2021. Journal: J Healthc Eng.

**Table 2:** Dataset description of proposed machine learning system.

Features	Description
M/F	Gender
Age	Person's age
EDUC	Years of education
SES	Socioeconomic status
MMSE	Mini-mental state examination
eTIV	Estimated total intracranial volume
nWBV	Normalized whole brain volume
ASF	Atlas scaling factor

**Table 3:** Comparison table of models.

Model	Accuracy (%)	Recall (%)	Precision (%)	AUC (%)	*F*1 score
SVM	92.0	91.9	91.9	91.9	91.9%
Logistic regression	74.7	70.3	76.5	74.6	73%.3
Decision tree	80.0	59.4	100	79.7	74.5%
Random forest	81.3	70.3	84.4	81.2	76.7%

## Data Availability

The data used to support the findings of this study are freely available at https://www.kaggle.com/jboysen/mri-and-alzheimers?select=oasis_longitudinal.csv.
